# The Human Homolog of Drosophila Headcase Acts as a Tumor Suppressor through Its Blocking Effect on the Cell Cycle in Hepatocellular Carcinoma

**DOI:** 10.1371/journal.pone.0137579

**Published:** 2015-09-10

**Authors:** Jun Wang, Li Gong, Shao-Jun Zhu, Qiao Zhu, Li Yao, Xiu-Juan Han, Jia-Rui Zhang, Yan-Hong Li, Wei Zhang

**Affiliations:** 1 The Helmholtz Sino-German Laboratory for Cancer Research, Department of Pathology, Tangdu Hospital, The Fourth Military Medical University, Xi’an, Shaanxi, China; 2 Department of Gynecology and Obstetrics, Tangdu Hospital, The Fourth Military Medical University, Xi’an, Shaanxi, China; University of Medicine, Greifswald, Germany, GERMANY

## Abstract

The molecular pathogenesis of hepatocellular carcinoma (HCC) is heterogeneous and extremely complex. Thus, for individual molecular targeted therapy, novel molecular markers are needed. The abnormal expression of the human homolog of Drosophila headcase (HECA homo) has been found in pancreatic, colorectal, and oral squamous cell carcinoma. Studies of oral squamous cell carcinoma have also demonstrated that the HECA homo protein can be negatively controlled by the Wnt-pathway and transcription factor 4 (TCF4) and can slow cell division by interacting with cyclins and CDKs. However, the role of HECA in HCC has not been reported elsewhere. Here, immunohistochemical analysis revealed that the downregulation of HECA homo protein occurred in 71.0% (66/93) of HCC cases and was positively correlated with a poorly differentiated grade, high serum AFP level, liver cirrhosis and large tumor size. The expression of HECA homo was detected in five live cell lines. In vitro, the overexpression of HECA homo in HepG2, Huh-7 and MHCC-97H cells could inhibit cell proliferation and colony formation and induce G1 phase arrest. In contrast, the downregulation of HECA homo could promote cell proliferation, colony formation and the cell cycle process. However, neither the overexpression nor downregulation of HECA homo in the three cell lines could affect cell migration or invasion. Collectively, HECA homo is regularly expressed in normal live cells, and the HECA homo protein level is heterogeneously altered in HCC, but the downregulation of HECA homo is more common and positively correlated with several malignant phenotypes. The HECA homo protein can slow cell proliferation to some extent primarily through its blocking effect on the cell cycle. Hence, the HECA homo protein may act as a tumor suppressor in HCC and might be a potential molecular marker for diagnostic classification and targeted therapy in HCC.

## Introduction

Hepatocellular carcinoma (HCC) is a major health problem worldwide, especially in Eastern and South-Eastern Asia, where 83% of the estimated 782,000 new cases worldwide are diagnosed, according to GLOBOCAN 2012. Notably, half of the new cases come from China, as more than 350,000 new cases are diagnosed yearly in China [1, 2]. Thus, the disease burden of HCC for China is great. Multiple risk factors for HCC exist in the environment and lead to the formation of a tumor microenvironment, including genetic and epigenetic alterations. In the molecular era, although substantial molecules, signal pathways and genetic profiling related to HCC have been found [3–5], to the best of our knowledge, none can be effectively applied for screening, early diagnosis, classification, targeted therapy, prediction of outcome or recurrence. The most essential reason for difficulty is that HCC is heterogeneous and evolving [5–7]. Even for an individual, a tumor is not static, and the corresponding molecular profiles are bound to vary over time over the disease course or treatment. Hence, the clinical application of molecular biomarkers for heterogeneous and evolving tumors, such as HCC, must be personalized, combined, and dynamically adjusted. To achieve this, the primary task is that more molecules related to the tumor should be identified.

Several reports have associated HECA homo with pancreatic [8], colorectal [9], and oral squamous cell cancer [10, 11]. Of note, all three of these tumor cell types, as well as HCC, originate from epithelial cells of the digestive system, which may share similar gene alterations. Thus, HECA homo may also be involved in HCC. In addition, studies on OSCC have confirmed that the overexpression of HECA homo could slow cell division [10]. Consistently, the silencing of HECA home could result in a significant increase in cell division and a markedly increased resistance against the chemotherapeutic cisplatin [11]. Furthermore, protein-protein interactions of HECA homo with CDK2, CDK9, Cyclin A and Cyclin K have been verified [11]. HECA homo expression can be suppressed by TCF4, which is a well-known Wnt-pathway-related transcription factor and can bind to the HECA homo promoter [11].

Moreover, HECA homo is a homolog to Drosophila HECA. Its influence on cell functions and the correspondent molecular mechanisms of HECA homo may be similar to those of Drosophila HECA. In Drosophila, HECA is critical for adult morphogenesis [12], such as the development of the trachea [13, 14], eye [15], and nervous system [16] and the maintenance of the stem cell niche in the testis [17]. Molecular mechanism studies have indicated that Drosophila HECA may be involved in the JAK/STAT [15] and Wnt pathways [18]. However, in humans, disorders of both JAK/STAT and Wnt pathways are involved in HCC [19], and abnormities of cell proliferation and differentiation are the most essential characteristics of any cancer.

From the perception of the molecular mechanism, cell function and tissue type, we possess ample and convincing evidence to presume that HECA homo has a certain antitumor function in HCC. Herein, to confirm the role of HECA homo in HCC, we examined the expression of HECA homo in HCC tissue samples and HCC cell lines and then analyzed the correlation between HECA expression and several clinicopathological features. We also separately up- or downregulated HECA homo expression in three HCC cell line to identify the possible effects of HECA homo on cell biological phenotypes.

## Materials and Methods

### Patients and tissue samples

Patients were selected from Tangdu Hospital (Xi’an, China) between January 2013 and December 2014, underwent a hepatectomy and were histopathologically diagnosed with HCC. Clinical and pathological data of all of the patients were collected. To compare the immunohistochemical results precisely and effectively, we selected a tissue mass with both tumor tissue and non-tumor tissue for each patient from our formalin-fixed and paraffin-embedded tissue bank. All of the procedures in this study were approved by the Research Ethics Committee of Tangdu Hospital. Written informed consent was obtained from all of the study participants.

### Immunohistochemistry (IHC)

Sections from paraffin-embedded tissues were immunostained with a rabbit polyclonal antibody for HECA homo (dilution: 1:200, Novus, Littleton, USA). Briefly, the activity of endogenous peroxidases was blocked with 3% H_2_O_2_ incubation for 15 min; heat-induced epitope retrieval was performed with 0.1 mol/l citrate buffer at pH 6.0. To avoid the interference of endogenous biotin, the MaxVision HRP-polymer anti-rabbit IHC kit (Maixin Ltd Company, Fuzhou, China) was applied. The sections were visualized through incubation with 3, 3’-diaminobenzidine (DAB) and then counterstained with hematoxylin. Normal human colon tissues were used as positive controls, and nonspecific IgG was used as a negative control.

### Immunohistochemistry assay

Each slide was independently examined by three pathologists through light microscopy. Usually, the granular brown color was recognized as positive immunostaining and can reflect the corresponding proteins. The scope of positive immunostaining reflects the location of the proteins. The intensity together with the scope of immunostaining can reflect the protein quantity. Here, we aimed to compare the protein quantity between two different cell types; thus, the protein quantity can be determined by immunostaining intensity without scope. Because tumor cells and paired non-tumor cells were on the same slide, it was easy to precisely determine the intensity difference. For each case, the HECA immunostaining intensity of tumor cells may be comparatively weak, equal, or strong compared with that of the adjacent non-tumor liver cells.

### Cell lines and cell culture

Cell lines, including HepG2, SK-hep-1, Huh-7, MHCC-97H and the normal human hepatocyte line HL-7702, were purchased from the cell bank of the Chinese Academy of Sciences. The cells were cultured in Dulbecco's modified Eagle's medium (DMEM, Hyclone, Logan, UT, USA), which was supplemented with 10% fetal bovine serum (Invitrogen, Carlsbad, CA, USA), 100 U/ml penicillin and 100 μg/ml streptomycin, and maintained in a humidified chamber at 5% CO_2_ and 37°C.

### Quantitative real-time PCR analysis (qRT-PCR)

The total cellular RNA was extracted from cells using the MiniBest universal RNA extraction kit (Takara, Dalian, China) and reversed transcribed by the PrimeScript 1st strand cDNA synthesis kit (Takara, Dalian, China) according to the manufacturer’s instructions. The cDNA was amplified using the QuantiFast SYBR Green PCR Kit (Qiagen, Hilden, Germany) on an ABI 7500 fast Real-Time PCR system (ABI, Foster city, CA, USA). The relative quantification was determined by the 2^-ΔΔ^Ct method. GAPDH mRNA was selected as an internal control. The specificity and purity of the PCR products were guaranteed by dissociation curves. The primers for HECA homo (forward: 5'-GGCTGCCTCTCCATGTTGT-3'; reverse: 5'-TGAGTCCTTCCACGATACCAA-3') and GAPDH (forward: 5'-GACAACAGCCTCAAGATCATCA-3'; reverse: 5'-TGAGTCCTTCCACGATACCAA-3') were purchased from Sangon Biotech (Shanghai, China).

### Western blot

The total cell protein was extracted, and the protein concentration was determined through a BCA assay (BeyotimeInc, China). A total of 40μg of total protein was loaded onto a 10% SDS-PAGE gel. The primary antibodies included mouse polyclonal antibody against human HECA (Abnova, Taiwan, 1:1000) and rabbit polyclonal antibody against β-actin (1:1000, Sigma-Aldrich, USA). The second antibody was an HRP-conjugated goat anti-mouse or goat anti-rabbit IgG (Santa Cruz Biotechnology, USA, 1:5000). An enhanced chemiluminescence reagent kit (GE Healthcare, USA) was used for visualization.

### RNA interference

To silence HECA homo expression, we used small-interference RNA (siRNA). A mixture of three predesigned siRNAs for HECA homo and a scrambled sequence as negative control were chemically synthesized (Genepharma, Shanghai, China). Transfection was performed by Lipofectamine 2000 according to the manufacturer’s recommendation. All of the siRNA sequences are presented in S1 Table. Three cell groups were set: siRNA group (mixture of three siRNAs targeting HECA homo), SNC group (scrambled siRNA as negative control) and blank group (Lipofectamine 2000 without any sequence). The effect of HECA homo silencing was confirmed by qRT-PCR and western blot analysis 48 h after transfection.

### HECA homo plasmid and transfection

A HECA homo open reading frame (ORF)-expressing clone containing a cytomegalomavirus promoter and the selectable marker for neomycin resistance was purchased from GeneCopoeia (Guangzhou, China). Transfections of cells were performed using Lipofectamine 2000 (Invitrogen, Carlsbad, CA, USA) according to the manufacturer’s instruction. Then, 24 h after transfection, the cells were subjected to geneticin (4 mg/ml) for at least two weeks to establish stable HECA homo-expressing clones. An empty pcDNA3.1+ plasmid from our lab was used as a mock control. Three cells groups were set: HECA exp group (cells transfected with HECA homo full-length-expressing plasmid), mock group (cells transfected with empty pcDNA3.1+) and blank group (cells treated only with Lipofectamine 2000). The effect of overexpressing HECA homo was tested by qRT-PCR and western blot analysis.

### Cell proliferation viability by MTT

The cell proliferation viability of the different processed cell groups was accessed by a 3-(4-,5-dimethylthiazol-2-yl)-2,5-diphenyl tetrazolium bromide (MTT) assay. In brief, 24 h after transfection, 200 μl of culture medium with 2000 cells was added to the single wells of 96-well plates in triplicate. Three identical plates were applied, and the absorbance of 450 nm was measured 24 h, 48 h and 72 h after inoculation.

### Wound healing assay

The migration ability of cells was accessed by a wound healing assay. Briefly, after the cell confluence reached approximately 90%, a linear scratch was made by a sterile micropipette tip. The scratch was photographed, and the width was measured at time points 0 h and 24 h from the same area. The migration ratio was calculated.

### Colony formation assay

Then, 24 h after transfection, 400 cells that were singly suspended were seeded onto a 60-mm plate and incubated for two weeks. Cell colonies were visualized by 1% crystal violet staining, and colonies with no less than 50 cells per single colony were counted.

### Cell invasion assay

An invasion assay was performed in a 24-well plate with Matrigel-coated polycarbonate filters with 8-mm pores (Corning Costar, USA). Briefly, 24 h after transfection, 1×10^5^cells with 200 μl of serum-free medium were seeded into the top chamber. The bottom chamber was filled with 200μl of medium containing 10% FBS. After 24 h of incubation, the cells of upper the chamber were removed by a cotton swab, and the cells below the chamber were fixed with methanol, stained with crystal violet and then counted by microscope in 10 random fields at ×200. For quantification, the average cell number per field for each membrane was calculated and is presented.

### Cell cycle and apoptosis analysis

The cell cycle and apoptosis were evaluated by flow cytometric analysis. In brief, 24 h after transfection, the cells were collected and fixed with 70% ethanol. Then, the cells were stained with a cell cycle detection kit or an Annexin V-PE/7-AAD apoptosis detection kit (Keygen, Nanjing, China) according to the manufacturer’s instructions. The data were collected and analyzed on a flow cytometer (Beckman-Coulter, Indianapolis, IN, USA) using the supporting software.

### Statistical analysis

The distribution of the original clinical data was examined using the Kolmogorov-Smirnov test. The data with a normal distribution are presented as the mean±SD (standard deviation). The data with a non-normal distribution are presented as percentiles. The correlation between variables was accessed by a Spearman rank correlation analysis. Three independent experiments were performed, and the values are presented as the mean±SD. The difference between two groups was assessed by an independent Student’s t-test, and the difference among three or more groups was assessed by a one-way analysis of variance. A two-tailed *p* value <0.05 was deemed significant. In all of the figures, * indicates *p*<0.05 and ** indicates *p*>0.05.

## Results

### Clinicopathologic features of HCC patients

A total of 93 patients with HCC were enrolled. The original information is presented in S2 Table. Generally, the ages were distributed normally (*p* = 0.524) and ranged from 27 to 79 years (mean: 51years). The male-to-female ratio was 6.75:1. Serum Hepatitis B surface antigen (HBsAg) was positive in 86.0% (80/93) of the patients. The serum alpha-fetoprotein (AFP) values were non-normally distributed (*p*<0.001) and ranged from 1.07 to 121000.00 ng/ml (25th percentile: 12.73, median: 253.70, 75th percentile: 3983). A total of 59.1% (55/93) of the patients had liver cirrhosis, and 63.5% (59/93) of the patients had a tumor with size of more than 5 cm in total diameter. Histopathologically, 11.8% (11/93) of the cases were well differentiated (Edmondson grade Ⅰ), 64.5% (60/93) of the cases were moderately differentiated (Edmondson grade Ⅱ), and 23.7% (22/93) of the cases were poorly differentiated (Edmondson grade III-Ⅳ).

### HECA homo protein level and location in HCC tissues

In all 93 cases, the HECA homo protein was present with consistent quantity in the non-tumor liver cells. Comparatively, the HECA homo protein in tumor cells was absent or present in a lower quantity in 71.0% (66/93) of the cases, present in an equal quantity in 21.5% (20/93) of the cases, and present in a greater quantity in 7.5% (7/93) of the cases. If detected, the HECA homo protein was exclusively located in the cytoplasm of liver cells. Representative pictures are presented in Fig 1.

**Fig 1:** Representative HECA homo protein immunohistochemical staining in HCC. The staining intensity of tumor cells is weaker than (A), equal to (B) or slightly stronger than (C) that of adjacent non-tumor cells. “T” indicates tumor area and “NT” indicates non-tumorous area. Magnification, ×100; scale bars, 100μm.

### Association of HECA homo protein quantity and clinicopathologic features

Statistical analysis showed that the HECA homo protein quantity was significantly correlated with the differentiation grade (r = -0.360, *p* = 0.000), serum AFP (r = -0.274, *p* = 0.008), cirrhosis (r = 0.243, *p* = 0.019) and tumor size (r = -0.224, *p* = 0.031). A decrease in the HECA homo protein quantity in tumor cells was likely in HCC patients with a poorly differentiated grade, high serum AFP level, liver cirrhosis or large tumor size. There was no significant association between the HECA homo protein and age, gender or HBsAg, as shown in Table 1. However, an exception could always exist for an individual.

**Table 1:** Association between the HECA homo protein quantity and clinicopathologic features of 93 patients with HCC.

Variants	n	HECA homo protein quantity		r^c^	*p* value
		T<N^a^	T≥N^b^		
All cases	93	66	27		
Age (years)				0.044	0.674
≤50	40	30	10		
>50	53	36	17		
Gender				-0.176	0.092
Male	81	55	26		
female	12	11	1		
Differentiation				-0.360	0.000
Well	11	2	9		
Moderate	60	45	15		
poor	22	19	3		
HBsAg				0.121	0.247
Negative	13	11	2		
Positive	80	55	25		
AFP (ng/ml)				-0.274	0.008
≤20	28	15	13		
≤400	22	18	4		
>400	43	33	10		
Cirrhosis				0.243	0.019
Absent	38	32	6		
Present	55	34	21		
Tumor size (cm)				-0.224	0.031
≤3	19	10	9		
≤5	15	11	4		
>5	59	45	14		

a: The HECA protein quantity of tumor cells is lower than that of adjacent non-tumor cells as detected by IHC

b: The HECA protein quantity of tumor cells is equal to or slightly greater than that of adjacent non-tumor cells as detected by IHC

c: Spearman rank correlation coefficient.

### Cell modes construction for altering HECA homo expression

HECA homo expression was detected at mRNA and protein level in all of the five cell lines. Ranked by the HECA homo expression level from high to low, the order was HepG2, HL-7702, Huh-7, SK-hep-1 and MHCC-97H (Fig 2A and 2D). We chose HepG2, Huh-7 and MHCC-97H cell lines for the following cell function assay. For each of the three cell lines, the knock-down of endogenous HECA homo was achieved by RNA interference, and the overexpression of HECA homo was achieved by the transient transfection of a full-length HECA-expressing plasmid. The efficiency of the knock-down or overexpression was confirmed at the mRNA and protein levels, respectively (Fig 2B, 2C and 2E).

**Fig 2:** Alteration of HECA homo expression in HCC cell lines detected by qRT-PCR and Western blotting. (A) The HECA homo mRNA level was the highest in the HepG2 cell lines among the five examined cell lines. (B) For each of the three cell lines (HepG2, Huh-7, and MHCC-97H), the HECA homo mRNA level in the siRNA group (cells transfected with specific siRNA against HECA homo) was significantly lower than in the SNC group (cells that were transfected with scrambled siRNA as a negative control) or in the blank group (cells treated with only Lipofectamine 2000). In contrast, there was no significant difference between the SNC group and the blank group. (C) The HECA homo mRNA level in the HECA exp group (cells that were transfected with HECA homo full-length-expressing plasmid) was significantly higher than those in the mock group (cells that were transfected with empty control plasmid) or blank group (cells that were treated with only Lipofectamine 2000). Meanwhile, there was no significant difference between the mock group and the blank group. (D) and (E) the corresponding protein levels were detected by western blotting.

### Effects of HECA homo on cell proliferation, clone formation, migration and invasion

Usually, tumor cell biological behaviors include proliferation, clone formation, migration and invasion. These behaviors can be assessed by MTT, colony formation, wound-healing and transwell invasion assays. The results based on the three cell lines (HepG2, Huh-7 and MHCC-97H) were similar. For each of the three cell lines, compared with cells that were transfected with the siRNA negative control, HECA homo knock-down cells exhibited increased proliferation and clone formation abilities (Fig 3) but no obvious alteration in the ability of migration or invasion (Fig 4). In contrast, compared with the cells that were transfected with empty plasmid, HECA homo-overexpressing cells showed decreased proliferation and clone formation abilities (Fig 3) but exhibited no obvious alteration in the ability of migration or invasion (Fig 4). The data indicate that HECA homo could play a role in cell proliferation and clone formation but not in cell migration or invasion.

**Fig 3:** HECA homo effects on HepG2, Huh-7, and MHCC-97H cells’ abilities of proliferation and colony formation. (A) Cell proliferation viability as assessed by MTT. For each of the three cell lines, the siRNA group exhibited more viability than did the SNC group, whereas the HECA exp group exhibited less viability than did the mock group. (B) Representative pictures for the cell colony formation assay (right) and quantitative analysis of colony number (left). For each of the three cell lines, more colonies were found in the siRNA group than in the SNC group, whereas fewer colonies were found in the HECA exp group than in the mock group.

**Fig 4:** HECA homo effects on HepG2, Huh-7, and MHCC-97H cells’ abilities of migration and invasion. (A) Representative pictures for the wound-healing assay (left, original magnification ×50) and quantitative analysis of the migration rate (right). For each of the three cell lines, the migration rate showed no significant difference between any of the groups. (B) Representative pictures of the transwell invasion assay (left, original magnification ×100) and quantitative analysis of invaded cells (right). For each of the three cell lines, there was no significant difference in the invaded cell numbers between any of the groups.

### Roles of HECA homo in the cell cycle and apoptosis

In fact, in a cell group, there are always some cells undergoing proliferation and some cells undergoing apoptosis or necrosis. To elucidate whether the effects of HECA homo on cell biological behaviors was due to its role in cell cycle regulation, apoptosis or necrosis, we examined the cell cycle and apoptosis by flow cytometric analysis in cell groups with different HECA homo expression levels. As shown in Fig 5A, for all of the three cell lines, the downregulation of HECA homo expression decreased the proportion of cells in G1 phase, and the overexpression of HECA homo increased the proportion of cells in G1 phase. Whereas neither downregulation nor overexpression of HECA homo in the three cell lines can affect the apoptosis rate, except that overexpressing HECA homo in HepG2 cells increased the apoptosis rate (Fig 5B).

**Fig 5:** HECA homo effects on cell cycle and apoptosis for HepG2, Huh-7, and MHCC-97H cells. (A) Representative pictures of cell cycle distribution as detected by flow cytometric analysis (left). Comparison of the relative cell numbers in the G1 phase between groups (right). For each of the three cell lines, fewer cells in the G1 phase were detected in the siRNA group than in the SNC group. And more cells in the G1 phase were found in the HECA exp group than in the mock group. (B) Representative pictures of apoptosis as detected by flow cytometric analysis (left). Comparison of the apoptosis rate (proportion of cells in early and late apoptotic stages) between groups (right). For each of the three cell lines, the apoptosis rate of the siRNA group was not significantly different from that of the SNC group, For Huh-7 and MHCC-97H cells, the apoptosis rate of the HECA exp group was also not significantly different from that of the mock group. But for HepG2 cells, the apoptosis rate of the HECA exp group was significantly higher than that of the mock group.

## Discussion

The limited application of molecular markers in the diagnosis and treatment of HCC mainly results from the heterogeneity of HCC. Tumor heterogeneity exists not only between patients but also between tumor nodules in the same patient and even within a single tumor nodule [5–7]. For an individual, a tumor is not static but is evolving, and the corresponding molecular profiles are bound to vary over time during the disease course or treatment. The heterogeneity is ubiquitous and determined by the diversity of environment and genetics. Therefore, it may be impossible to find a molecular maker that is wildly applicable for diagnosis or treatment for most HCC patients. However, for an individual, molecular markers can be used for risk stratification and can be developed for individual targeted therapy; thus, more molecules should be prepared.

In normal human tissues, HECA homo is ubiquitously expressed at a basal level, with the highest expression in the spleen, prostate and peripheral blood leukocytes [8]. In the present study, the HECA homo protein was regularly expressed in normal live cells and was located in the cytoplasm. The downregulation of HECA homo protein was frequent (71.0%), especially in HCC patients with a poorly differentiated grade, high serum AFP level, liver cirrhosis or large tumor size, all of which are indicators for the poor prognosis of HCC patients. The normal regulation or even upregulation of the HECA homo protein level was also present in some patients (29.0%).

These results indicate that HECA homo expression is heterogeneously changed during HCC progression. For HCC patients, the downregulation of the HECA homo protein may promote HCC development, but this protein is not indispensable since HECA homo protein was not downregulated in all of the cases. The upregulation of HECA homo may slow HCC progression, but its antitumor effect could be neutralized by other oncogenic effects. And the upregulation of the HECA homo protein may be the compensatory reaction of cells to counteract other oncogenic factors. Hence, it is not surprising to find that there were some HCC patients with upregulated HECA homo expression even it is a tumor suppressor.

There is also the possibility that the HECA homo protein has no effect on the malignant phenotypes of tumor cells, such as proliferation, migration or invasion. The alteration of the HECA homo protein level may only be a passing alteration during tumor progression, because the alterations caused by risk factors are usually nonspecific at the molecular level. For example, DNA mutation is one of the most important mechanisms that lead to tumors, but in HCC, mutations caused by the HBV virus, oxygen-free radicals or aflatoxin are usually nonspecific to genes. If a gene is functionally mutated with a high frequency among a tumor group, we can only conclude that the gene is prone to being injured. And this gene may be a potential diagnosis marker with high sensitivity for this tumor type. However, we cannot conclude that the functional disorder of this gene is indispensable for tumor formation or that the disorder of this gene in a cell would change the cell to a tumor cell. Therapy targeting this gene may thus be invalid. Moreover, the HECA homo protein level as detected by IHC at a time point is a reflection of a dynamic balance between HECA homo protein synthesis and degradation. Both protein synthesis and degradation are extremely complex processes that involve many genes and related molecules that can be genetically or epigenetically changed. In addition to HECA homo itself, any heritable change in related genes in the system can alter the HECA homo protein level.

However, regardless of the mechanisms through which the HECA homo protein level can be changed during HCC progression, as long as we can confirm that the HECA homo protein associates with some malignant phenotypes of a tumor cell, this protein could be a potential therapy target. Therefore, to further identify the role of HECA homo in HCC, we upregulated or downregulated HECA homo expression in HepG2, Huh-7 and MHCC-97H cells. For all of the three cell lines, cell function studies have indicated that HECA homo could play a role in cell proliferation and clone formation but not in cell migration or invasion. The upregulation of HECA homo suppressed cell proliferation and colony formation, whereas the down regulation of HECA homo promoted cell proliferation and colony formation. Further studies of the cell cycle indicated that, for all of the three cell lines, the upregulation of HECA homo increased the proportion of cells in G1 phase, whereas the downregulation of HECA homo decreased the proportion of cells in the G1 phase. Studies of the apoptosis indicated that neither upregulation nor downregulation of HECA homo could significantly change the apoptosis rate for the three cell lines, except that upregulation of HECA homo in HepG2 cells increased the apoptosis rate.

In fact, in vivo, the migration and invasion of tumor cells are closed related to the proliferation of tumor cells. However, in migration and invasion studies in vitro, the effect of cell proliferation was suppressed artificially; therefore, it was not surprising that HECA homo could play a role in cell proliferation but not in cell migration or invasion in vitro. In addition, the effects of the HECA homo protein in cell cycle control and the corresponding molecular mechanism have been reported in studies on oral squamous cell carcinoma [10, 11]. These results strengthen our hypothesis that HECA homo acts as a tumor suppressor in HCC.

However, to date, not all studies have indicated that HECA homo acts as a tumor suppressor. Consistent with our findings, studies on pancreatic cancer and oral squamous cell carcinoma have indicated that HECA homo expression is prone to decrease or become lost in cancer cells [8, 10, 11]. In contrast, one study on colorectal cancer indicated that HECA homo expression was upregulated in blood and fecal samples of patients, especially in early stage colorectal cancer [9]. There are several possible explanations for these inconsistent findings. The difference may result from differences in the elements in each study, such as experimental technologies, sample types, cancer types, and population race. In addition, HECA homo may have an antitumor effect in colorectal cancer because the upregulation of HECA homo expression in patients might be the compensatory reaction of our body to oncogenic factors. Of course, further studies including more clinical samples with detailed information and studies on the molecular mechanisms and animal mode are needed to confirm the antitumor role of HECA homo in HCC or other tumor types.

In summary, we are the first to report the role of HECA homo in HCC. HECA homo is regularly expressed in normal live cells and is heterogeneously altered during HCC progression. The downregulation of the HECA homo protein in HCC is common and positively correlated with several malignant phenotypes. The HECA homo protein can slow down cell proliferation to some extent primarily through its blocking effect on cell cycle. Thus, the HECA homo protein may act as a tumor suppressor in HCC and might be a potential molecular marker for diagnostic classification and targeted therapy in HCC.

## Supporting Information

S1 Table Information of siRNAs. (DOCX)

S2 Table Clinicopathological data and HECA homo protein as detected by IHC in 93 HCC patients. (DOCX)
